The article "Molecular Mechanism Underlying Lymphatic Metastasis in Pancreatic Cancer" was published in 2014. Journal: Biomed Res Int.

# Molecular Mechanism Underlying Lymphatic Metastasis in Pancreatic Cancer

**DOI:** 10.1155/2014/925845

**Published:** 2014-01-22

**Authors:** Zhiwen Xiao, Guopei Luo, Chen Liu, Chuntao Wu, Liang Liu, Zuqiang Liu, Quanxing Ni, Jiang Long, Xianjun Yu

**Affiliations:** ^1^Department of Pancreatic and Hepatobiliary Surgery, Fudan University Shanghai Cancer Center, Shanghai 200032, China; ^2^Department of Oncology, Shanghai Medical College, Fudan University, Shanghai 200032, China; ^3^Pancreatic Cancer Institute, Fudan University, No. 270, Dong'An Road, Xuhui District, Shanghai 200032, China

## Abstract

As the most challenging human malignancies, pancreatic cancer is characterized by its insidious symptoms, low rate of surgical resection, high risk of local invasion, metastasis and recurrence, and overall dismal prognosis. Lymphatic metastasis, above all, is recognized as an early adverse event in progression of pancreatic cancer and has been described to be an independent poor prognostic factor. It should be noted that the occurrence of lymphatic metastasis is not a casual or stochastic but an ineluctable and designed event. Increasing evidences suggest that metastasis-initiating cells (MICs) and the microenvironments may act as a double-reed style in this crime. However, the exact mechanisms on how they function synergistically for this dismal clinical course remain largely elusive. Therefore, a better understanding of its molecular and cellular mechanisms involved in pancreatic lymphatic metastasis is urgently required. In this review, we will summarize the latest advances on lymphatic metastasis in pancreatic cancer.

## 1. Introduction

Pancreatic adenocarcinoma (PDAC) is notorious for its abysmal propensity of early lymphatic invasion, liver metastasis, recurrence, and poorest prognosis. Less than 5% of patients will live up to 5 years once diagnosed [1]. The radical surgery, as yet, is the sole way of possibility to achieve long-term survival for resectable patients with this disease. Lymphatic metastasis, including micrometastases in lymph node, is an early adverse event and independent poor prognostic factor of resected PDAC patients. According to a large population-based retrospective study [2], patients without lymph node metastasis (N0) had a notably better overall survival than those with nodal disease (N1) (median survival, 18 months versus 12 months). Moreover, the incidence of lymphatic metastasis in PDAC is very high, approximately 65.3 to 89%, even in cases with small tumors less than 2 cm [3, 4]. Worse still, about 40% of the negative lymph nodes in conventional histopathology can be redetected by specific immunohistochemistry or PCR analysis as positive for micrometastases and nodal micrometastases occurred in 75% around N0 patients [4–6]. Therefore, to terminate the double high features of PDAC, namely, high mortality and high metastasis rate, is the critical step to lower mortality of this refractory disease.

The article "Molecular Mechanism Underlying Lymphatic Metastasis in Pancreatic Cancer" was published in 2014. Journal: Biomed Res Int.

Generally, lymph node metastasis would not directly cause fatal damage to patients, but rising evidence revealed that the disseminated cancer cells in lymph node may be the driver of relapse in local and distant organs that result in the death of patients in the end. Classically, lymphatic metastasis often includes six steps, namely, detachment from the original tumor, locomotion into the matrix, anchoring the lymphatic vessels, surviving in the circulation, settling in a hospitable site of lymph nodes, and colonizing to form mature metastases [7]. But in actual fact, the evolution of this process, far from these steps, is more dynamically undergoing subtle alteration of the cancer cells themselves synergized with modeling of the tumor microenvironment and the premetastatic sites (or niche). Analogous to other styles of metastasis, three conditions are necessary for lymphatic metastasis: one is the ability of cancer cells to obtain higher immigrating invasiveness, that is, the formation of MICs; another is the well-prepared milieus or niche suitable for tumor growth and dissemination; and last is the chemoattractants released by cancer cells or interstitial cells, these have a guiding role in organ-specific metastasis of MICs. Of note, the metastatic lesions in lymph nodes may be a “seed reservoir” for metastatic formation in distant organs via lymphatico-venous communication. The lymph node metastases not only serve in a direct or indirect role for the systemic metastases but also indicate an invasive phenotype of cancer cells.

Herein, the most formidable challenge we are now confronted with is how to nip the metastases in the bud or improve the early diagnosis of PDAC patients. Undoubtedly, an improved understanding of the mechanism underlying lymphatic metastasis in PDAC is necessary to combat this daunting disease. In this review, we will summarize the molecular and cellular mechanisms of lymphatic metastasis in PDAC, aiming to explore the corresponding targeted therapeutic strategies along with our institution's experiences.

## 2. Cellular and Molecular Events Underlying Lymphatic Metastasis in Pancreatic Cancer

### 2.1. CSCs and MICs

As the “roots” of the metastases, MICs play a critical role in lymphatic metastatic dissemination. Emerging evidence indicates that cancer cells are not a pure homogenous group but constituted by a cluster of heterogeneous cancer cells containing cancer stem cells (CSCs), MICs, and others [8–11]. The existence of CSCs was originally verified by a small population of leukemia cells obtained from patients. When implanted into immunodeficient mice, they would develop into an identical new tumor [12]. Afterwards, the eyes of some scholars were turned to solid tumors and intriguingly found that a small subset of cancer cells isolated from solid tumors were also able to generate new tumor in xenograft mice model and endowed with the capacity of serial passage, sphere-formation, and self-renewal in vitro as well [9, 13]. Moreover, regarding CSCs the apexes of the cancer cell groups that is not a homogenous population either, play diverse roles in tumorigenesis and progression depending on their various phenotypes (Table 1) [8, 9]. MICs, a subpopulation of CSCs, acquired the same somatic mutations as CSCs but are epigenetically distinct; not only do MICs possess the phenotypes of self-renewal, tumor initiation, and tumor propagation, but are also responsible for initiating tumor metastases (Figure 1) [9, 10]. To the best of our knowledge, the MICs play a critical role in lymph node metastasis for pancreatic cancer though they account for only a small part of pancreatic cancer cells, less than 1–5% of total cancer cell population [13–15].

The article "Molecular Mechanism Underlying Lymphatic Metastasis in Pancreatic Cancer" was published in 2014. Journal: Biomed Res Int.

Of the various known stem markers for CSCs (Table 1), only a few are specifically linked to metastasis. Hermann and his colleagues investigated that only CD133^+^CXCR-4^+^ pancreatic CSCs were capable of driving metastasis through orthotopical injections into athymic mice; in contrast, CD133^+^CXCR-4^−^ stem cells are limited to developing primary tumors with less or no metastases [9]. But a profound analysis had been made to the specimens resected from 80 patients with PDAC demonstrating that CD133^+^ expression had a significantly positive correlation with lymphatic invasion regardless of whether there existed CXCR-4 expression or not [14]. However, there is evidence that CXCR-4 can induce de novo lymphangiogenesis and angiogenesis within the tumor or secondary site in pancreatic cancer, which may be favorable for lymphatic invasion [16]. Anyway, the discrepancy in their investigations is not beyond our expectation to some degree because of the complexity and variance of human pancreatic cancerous tissues compared with xenograft models. The expression of the CXCR-4 receptor on tumor cells is just a novel marker correlated with poor survival and high lymphatic invasion rate of pancreatic cancer [16, 17], but not the checkpoint of lymphatic metastasis. Therefore, we may speculate that the determinants of lymph node metastasis are polyphyletic, including the quality of the cancer cell itself, tumor microenvironment, and niche.

The article "Molecular Mechanism Underlying Lymphatic Metastasis in Pancreatic Cancer" was published in 2014. Journal: Biomed Res Int.

### 2.2. Gene Alteration

Gene alteration or gene instability is the intrinsic cause of tumor pathogenesis and metastatic dissemination including lymphatic metastasis and is intensely linked with the evolvement of cancer cells into CSCs or MICs as well. Currently, there are two hypotheses about tumorigenesis [18]: the most classical one is gene mutation, which highlights that the initiation and progression of tumor are caused by accumulating different gene mutations; while in contrast, another increasingly popular hypothesis, genome aneuploidy, is conceived to be the main determinant of tumorigenesis and tumor progression. Through our previous participating research, we found that gene susceptibility had an intense correlation with pancreatic cancer initiation. We observed that five new susceptibility loci at chromosomes 21q21.3, 5p13.1, 21q22.3, 22q13.32, and 10q26.11 are significantly associated with pancreatic cancer risk in Chinese populations [19]. Furthermore, we have established a cell line BxPC-3-LN derived from cell line BxPC-3, possessing high capacity of lymphatic metastasis (Figure 2). And interestingly, we observed that some metastasis-related genes expression was significantly distinct from that of the parental BxPC-3. For instance, MMP14, MMP24, MIF, R-RAS, and ADRM1 were significantly overexpressed, while the genes such as TGFB2 and ROBO1 were prominently downregulated compared with those of parental BxPC-3 by global gene microarray [20]. However, the more direct evidence is that several animal models of pancreatic cancer have been established employing genetic engineering technique. KRAS mutation, as a popular phenomenon in pancreatic cancer patients, has been applied mostly the establishment of animal model. This gene mutation is mainly related to the pancreatic intraepithelial neoplasia but rarely lead to invasive PDAC. Nevertheless, it is strikingly found that when integrated with deficient Ink4a/Arf, the engineered mouse with activated KRAS would suffer from metastatic PDAC [21]; similarly, when combined with mutation p53 rather than deficiency p53, the activated KRAS would also give birth to new metastases in PDAC; in addition, p53 accumulation was significantly correlated with lymph node metastasis [22, 23]. And two recent novel researches [24, 25] indicated that the metastases were the results of cancer cells with genetic heterogeneity within primary tumor, some of which were capable of triggering metastasis. And they further declared that some mutated genes (CNTN5, DOCK2, MEP1A, and LMTK2) or rearrangements were just found in index metastatic lesions from these patients with Stage IV disease instead of in the primary pancreatic index lesions. The primary tumor of PDAC containing a mix of geographically distinct subclones contributed greatly to the formation of different metastases separately. And all indications are that the evolution of genetic clone within primary tumor may be the real culprit of metastases. Mountings of studies have revealed that some genes' aberrant expression had a significant correlation with the lymphatic metastasis of pancreatic cancer via global genomewide cDNA microarray assay [26, 27]. Kim et al. found that the expressions of genes such as SCA1, TNFRSF5, and SIX1 were significantly upregulated in pancreatic cancer patients with lymph node metastasis, while those of CAMKK2, GADD45A, ATF3, SLIT2, SPRY2, CTNNB1, CDH19, and TLN2 were obviously downregulated, and further presumed that they might contribute to the process of lymph node metastasis by involvement of apoptosis, cell cycle, cell growth, cell adhesion, and motility [26]. Nakamura and colleagues also sifted 76 candidate lymphatic metastasis-related genes such as RPS15A, RPA2, USP22, TMEPAI, and HADHA [27]. Although no one gene has been validated to be the cause of lymphatic metastasis, we could scrupulously extrapolate that gene alteration or gene instability may contribute to this process in some way.

The article "Molecular Mechanism Underlying Lymphatic Metastasis in Pancreatic Cancer" was published in 2014. Journal: Biomed Res Int.

Lymphatic metastasis is conceived of the synergistic result of accumulative gene alteration of cancer cells and adaptive change of tumor-supportive microenvironment. Recent data showed that more than 5 years were required for the development of metastatic subclones within nonmetastatic parental tumor after its formation, and another 1–3 years were needed for these clones to spread to specific second organs and cause patient death [24]. Taken together, we could prudently recapitulate that the metastases including lymphatic metastasis may seem to be an early event due to high incidence of lymph node metastasis in pancreatic cancer patients but in reality a late event in clonal evolution of this disease. Therefore, it might provide a large window of opportunity for early diagnosis of pancreatic cancer via detection of cancer-related genes.

### 2.3. Micro-RNAs

Micro-RNAs (miRNAs) as a family of single-stranded, evolutionarily conserved, endogenous, and small noncoding RNA molecules constituted of 22 nucleotides around, often function as posttranscriptional gene regulators involved with diverse physiological and pathophysiological functions. Recent evidence indicates that miRNAs are capable of acting as antioncogenes and oncogenes in tumorigenesis and progression of PDAC [32]. As further research conducted on miRNAs, more metastasis-related miRNAs are discovered at full speed, whereas the association between miRNAs and lymph node metastasis is infrequently reported in PDAC. Our recent study on miRNAs profile of high lymph node metastatic cell line BxPC-3LN revealed that some miRNAs were significantly down- or unregulated compared with that of parental BxPC-3 (data not published), and intriguingly we found that some of their target genes predicted by some target software (TargetScan Human, miRWalk, and miRecords) were well consistent with our previously reported gene array data (Figure 2) [20].

The article "Molecular Mechanism Underlying Lymphatic Metastasis in Pancreatic Cancer" was published in 2014. Journal: Biomed Res Int.

The link between miRNAs and metastasis in multiple malignancies including PDAC is reported to be the ability of some miRNAs to epigenetically modulate metastasis-related gene expression and vital molecules of signaling pathways. Tavano and colleagues [33] had made an analysis of correlations between changes of miRNA-143 and miRNA-21 expression and clinicopathological of PDAC patients indicating that miRNA-143 expression was negatively related to lymph node metastasis. However, they did not unravel the definite mechanism between them until now. Kent et al. [34] observed that miRNA-143/145 cluster were frequently repressed in KRAS mutant pancreatic cancers animal model, meanwhile, restoration of these miRNAs could abrogate tumorigenesis. They further found that repression of miRNA-143/145 cluster could trigger a tumor-promoting feedforward pathway by targeting KRAS and Ras-responsive element-binding protein (RREB1). KRAS gene has been reported to be a target of multiple miRNAs in PDAC. MiRNA-96 could directly downregulate the KRAS oncogene to restrain cancer cell invasiveness and immigration [35]. MUC4 was verified to be highly expressed in PDAC and reversely related to prognosis [36, 37]. Choudhury and colleagues observed that PDAC with high MUC4 expression showed a significant relevance to metastases of distant lymph nodes and faster tumor growth compared to those with MUC4 low expression in vivo [37]. MiRNA-150 mediated downregulation of MUC4 expression leading to reduced activation of downstream signaling and then suppressing the growth, invasion, and metastasis of pancreatic cancer cells [36]. Moreover, some tumor-suppressive miRNAs could directly or indirectly influence stemness of cancer cells to inhibit tumor metastasis. The downregulation of miRNA-200 family can promote metastasis and tumor-initiating capacity of pancreatic cancer cells by targeting ZEB1 and stem cell factors, such as Sox2 and Klf4 [38]. Another novel study indicated that miRNA-34 also had an impact on stemness of pancreatic cancer cells potentially by targeting Bcl-2 and Notch1/2. It may retrieve the tumor suppressing function of the p53 in p53-deficient human pancreatic cancer cells [39].

The article "Molecular Mechanism Underlying Lymphatic Metastasis in Pancreatic Cancer" was published in 2014. Journal: Biomed Res Int.

In contrast, miRNAs regarding having another role in oncogenic function are, likewise, important in invasiveness and metastasis of PDAC. Numerous studies demonstrated that miRNA-10a and miRNA-10b were markedly overexpressed in pancreatic cancer cells and further verified that miRNA-10a promoted the invasive ability of cancer cells partially via suppression of HOXA1, HOXB1, and HOXB3 genes [40, 41]. They observed that expression of miRNA-10a, as a retinoid acid target was effectively repressed by retinoic acid receptor antagonists. And simultaneously, the metastasis behavior of pancreatic cancer cells was completely blocked [41]. Inhibition of miRNA-27a suppressed the growth, colony formation, and migration of pancreatic cancer cells, and further data indicated that miRNA-27a played an oncogenic role and modulated the malignant, biological behavior of pancreatic cancer cells by targeting SPRY2 [42].

### 2.4. Molecular Signal Pathways

The molecular signal pathways are extensively involved in the initiation and progression of PDAC. However, little information has been clarified on their role in lymphatic invasion of this intractable disease. Herein, we mainly focus our attention on their function to enhance metastatic ability of cancer cells and how they direct the dissemination of tumor cells to peripheral lymph nodes.

TGF-beta signal axis plays a paradoxical role in pancreatic cancer as either a tumor suppressor or promoter mainly depending on its downstream effectors. TGF-beta exerts its significant impact on anticancer mainly in Smad-dependent manner (TGF-beta/TGF-betaRI/II-Smad2/Smad3-Smad4-Targeted genes-Anticancer), which can be negatively modulated by Smad7 and Smurfs [43]. Multivariate analysis based on pancreatic cancer patients showed that low-level Smad7 and Smad4 expression had shown a significant negative correlation with lymph node metastasis [44, 45], while TGF-beta, playing a distinct role in PDAC pathogenesis, can mediate tumor promotion or a more aggressive phenotype attributing its effect on tumor cell and tumor-supportive microenvironment. TGF-beta could modulate epithelial mesenchymal transition (EMT-) associated gene expression, leading to reduction of E-cadherin and increased expression of Snail and Matrix Metal Proteinase-2 (MMP-2) [46]. The overexpression and activation of MMP-2 have an adverse correlation with distant lymph node metastasis integrated with the expression of integrin alphaVbeta3 of pancreatic cancer cells [47, 48].

Clinical evidence reveals that aberrant expression of Sonic Hedgehog (Shh) is tightly correlated with TNM of PDAC patients [49]. Shh inserts its protumor effect in PDAC principally by promotion of desmoplasia, EMT evolution, and acquisition and maintenance of stemness of CSCs. Experimentally, Hedgehog/Gli signal allied with epidermal growth factor receptor (EGFR) signaling promoted transformation and cancer cell proliferation in vitro and in vivo by activation of HH-EGFR cooperation response genes including SOX2, SOX9, JUN, CXCR4, and FGF19 and further suggested that it was necessary for growth and maintenance of CSCs [50]. A recent study showed that Gli1 synergized with TGF-beta may induce an EMT phenotype contributing to the highly metastatic phenotype of PDAC [51]. The activation of HH signaling cascade can drive desmoplasia in PDAC and indicated an ominous prognosis [52].

The article "Molecular Mechanism Underlying Lymphatic Metastasis in Pancreatic Cancer" was published in 2014. Journal: Biomed Res Int.

Notch, known as a transmembrane receptor that mediates local cell-cell interaction, in mammals, which consists of four distinct subtypes Notch-1, Notch-2, Notch-3, and Notch-4, and nearly all of them are functioned in ligand-dependent manner, the canonical ligands such as delta-like and jagged, as well as other noncanonical ligands like F3/contactin [53]. Dysregulation of the Notch signaling pathway is frequently observed in human cancer including pancreatic cancer and predicts an invasive phenotype [11, 54]. Recently, an elegant study analyzing surgical specimens of PDAC showed that high Delta-like 4 expressions were independently related to both advanced tumor stage and lymph node metastasis [55]. And there are proofs indicating that overexpression of Notch-1 induced EMT phenotype and increased properties of CSCs by activation of mesenchymal cell markers such as ZEB1, Hes-1 and modulation of metastasis-related miRNAs such as miRNA-21, miR-200, and let-7 family members (Table 2) [56, 57]. However, a disparate viewpoint proposed that Notch-1, as a tumor suppressor in pancreatic cancer, was verified in a model of KRAS-induced PDAC [58]. Furthermore, aberrant expression of Notch induced by MMP-7 and ADMA metalloproteinase conjunct with KRAS mutation can prompt rapid reprogramming of acinar-to-ductal metaplasia (ADM), which has been hypothesized to play cardinal role in the evolvement of pancreatic cancer [59, 60].

The chemotaxis of signal pathways in lymphatic metastasis of PDAC is recently well studied. Compelling evidence revealed that SDF-1/CXCR-4 signal axis was important in the progression and metastatic dissemination of PDAC, especially well known for its recruitment of cancer cells to specific organs. CXCR-4 has been proven to be expressed in pancreatic intraepithelial neoplasia (PanIN), PDAC, and especially the metastatic site playing a crucial role in lymphangiogenesis [16] and regulation of tumor cell proliferation, metastasis, and chemoresistance [17, 67–70]. Recent evidence has shown that it mediated site-specific metastasis of pancreatic cancer cell to the liver and lung in an engineered mouse model [71]. More interestingly, it has also been identified that SDF-1/CXCR-4 axis has a significant correlation with lymph node metastasis in PDAC [16] and other tumors such as breast cancer, colorectal cancer, and gastric cancer [72–74]. Cui et al. investigated in PDAC specimens that high expression of SDF-1 was detected in paracancerous tissues, normal pancreas, and lymph nodes in contrast with lower expression in tumor tissues, while the distribution of CXCR-4 expression showed an opposite trend. Meanwhile, they observed that the expression of CXCR-4 has a significant association with microlymphatic vessel density (MLVD) and the lymph node status of PDAC patients. Taken together, they deduced that SDF-1/CXCR-4 may interact in ligand-receptor style leading to chemotaxis that SDF-1 would direct CXCR-4 positive cancer cells to lymph nodes with high concentration of SDF-1 [16]. Further studies into metastatic mechanisms showed that SDF-1/CXCR-4 could modulate proliferation and progression of pancreatic cancer cells through CXCR-4-dependent activation of signal pathways, such as MAPK/ERK1/2, PI3K/Akt, FAK, Src, and STAT, which plays a core role in its devastating behavior [75–77]. In addition, SDF-1/CXCR-4 signal axis functions as an essential messenger for “homing” of myeloid-derived cells to the primary tumor and the metastatic site or niche [78]. Thus, SDF-1/CXCR-4 may contribute greatly to the formation of tumor microenvironment and niche. CXCR-4 is highly expressed in MICs and indicative of invasive phenotype. Additionally, taking the distinct distribution of SDF-1/CXCR-4 in the main sites of pancreatic cancer metastasis [9, 16] and significant depressive effect on tumor migration interfered by CXCR-4 antagonist and such as shRNA, AMD3100, and TN14003 [31, 79] into consideration, the signal axis of SDF-1/CXCR-4 is crucial for the lymphatic metastasis of pancreatic cancer.

The article "Molecular Mechanism Underlying Lymphatic Metastasis in Pancreatic Cancer" was published in 2014. Journal: Biomed Res Int.

Of the same family, CCR7 combined with its ligand CCL21 was recently reported to synergistically guide pancreatic cancer cells toward lymphatic vessels and promote lymph node metastasis [80, 81]. Shields and his coworkers creatively verified in a 3-dimensional model that CCL19/CCL21-CCR7 axis mediated an autologous chemotaxis to the lymphatics via interstitial flow and gradient-dependence of autocrine CCL19/CCL21; and interestingly, further research revealed that interstitial flow-enhanced migration cannot be reduced by blockage of CCR7, which implicated that direct proteolysis may be the main cause of flow-enhanced migration in that it can be abolished by pan-MMP inhibitor GM6001[82]. Based on the above research, William and his group observed that flow-enhanced guided migration could be competed by CCR7-independent mechanism. This hypothesis could be supported by the experimental data that decreasing cell density could reverse the directional bias of migration. In vivo, Sperveslage and colleagues demonstrated that CCR7 transfected PT45P1 cells orthotopically injected in nude mice produced significantly larger tumors and exhibited a higher frequency of lymph vessel invasion and lymph node metastases compared with mock transfected cells. And the expression of CCR7 and its ligands CCL19/CCL21 in human pancreatic cancer tissue had an obvious correlation with the high rate of lymphatic metastasis [81]. Issa et al. led an elegant research showing that expressions of VEGF-C and CCR7 by tumor cells synergistically directed themselves toward lymphatics via increasing CCL21 secreted by lymphatic endothelial cells [80]. The effect on lymphatic metastasis of CCL19/CCL21-CCR7 axis was also observed in other tumors [82, 83].

VEGF-C/-D, the members of VEGF family, were deemed as specific lymphangiogenic growth factors, together with their cognate receptors EGFR-2/3, which have attracted a wide range of concern on the role of tumor-associated de novo lymphangiogenesis and lymphatic metastasis [80, 84]. VEGF-C and VEGF-D precursors, as pre-pro-polypeptides, which have low affinities with EGFR-2/3, to increase their affinities and implement their biologic function efficiently, are in need of stepwise proteolytic processing to become mature VEGF-C and VEGF-D/a central VEGF homology domain (VHD) [85, 86]. Therefore, theoretically, any factors influencing their affinities and output would disturb the lymphangiogenesis and lymphatic metastasis. One study after another indicated that high expression of VEGF-C or VEGF-D in a variety of tumors including pancreatic cancer had a significantly high incidence of lymph node metastasis [84, 87]. In contrast, there were no statistical correlations between expression levels of VEGF-C or -D and liver metastasis [84]. However EGFR-2 and -3 have been reported to be expressed in vascular endothelium but not on malignant cells, and they may insert a certain role in regulating de novo angiogenesis and lymphangiogenesis within tumor or premetastatic foci [88, 89]. EGFR-3 expressed on lymphatic endothelial cells which can bind with VEGF-C/D secreted by both pancreatic cancer cells and tumor-associated macrophages (TAMs) results in tumor lymphangiogenesis and chemoattraction of tumor cells toward lymphatic endothelial cells (LECs) [80, 84, 90]. However, the axis of VEGF-C/-D/EGFR-3 is modulated by many other factors such as Ang-1/2, Tie2, and integrins. Accordingly, these provide us with a new insight into overcoming this devastating event that not just targeting some molecules.

The article "Molecular Mechanism Underlying Lymphatic Metastasis in Pancreatic Cancer" was published in 2014. Journal: Biomed Res Int.

## 3. Lymphangiogenesis and Lymphangiogenic Factors

Much progress has been made in the angiogenesis and the growth of blood vessels over the past few decades, while less is known about the lymphangiogenesis. In recent years, substantial progress has been made in the identification of a series of specific lymphatic markers and regulatory molecules, which have provided a feasible way insight into the relationship between tumor lymphangiogenesis and lymphatic metastasis.

Generally, the lymphangiogenesis follows two pathways including embryonic and sprouting styles. The embryonic lymphangiogenesis, at about embryonic 7 weeks in humans or about embryonic 10 days in mice, starts to germinate from a specific cardinal vein that highly expresses VEGF-3, accompanied with changes in expression of some related genes and lymphangiogenic factors, for instance, LYVE-1, SOX18, Prox1, Neuropilin-2, Spred-1/-2, podoplanin, Syk, SLP-76, PLC-gamma, FoxC2, NFATc1, and ephrinB2; in concert with these changes, the cardinal vein gradually undergoes differentiation, intrinsic remodeling, and at last maturation into functional lymphatic vessels [91]. Alternatively, sprouting lymphangiogenesis is in some part distinct from the former. It mainly sprouts from the preexisting lymphatic vessel, and with the cooperation of recruiting lymphatic endothelial progenitor cells, mesenchymal precursors, lymphatic angioblasts, and other sources of lymphatic endothelia cell, to develop the primary lymphatic plexus, which are subsequently remodeled into hierarchal lymphatic. While the neoplastic lymphangiogenesis is widely thought to follow through the latter approach, but the lack of some remodeling and maturation related molecules, the neoplastic lymphatic vessels are oftentimes in malfunction and chaos, particularly those inside tumor. Therefore, some scholars conceived that the lymphangiogenesis inside tumor does not play a role in lymphatic invasion and only those occurring in paratumor may contribute to lymph node metastasis in pancreatic cancer [92]. However, research led by Cao et al. suggested that PDGF-BB enables promotion of pancreatic cancer lymphatic metastasis partly by inducing intratumoral lymphangiogenesis [93]. Similar cases are reported by Lee's [94] and He's groups [87]. Considerable data supports that lymphangiogenesis acts as a co-conspirator with cancer cells dispersing to lymphatic circulation in the lymphatic metastasis event of PDAC [16, 95]. The de novo lymphatic characterized with no continuous basement membrane, lacking pericyte and tight interendothelial junctions, provides an advantaged ductus network for tumor cells to penetrate into lymphatic vessel. Furthermore, EGFR-3 expressed on lymphatic endothelial cells which can bind with VEGF-C/D secreted by both pancreatic cancer cells and tumor-associated macrophages (TAMs) results in tumor lymphangiogenesis and chemoattraction of tumor cells toward LECs [84, 90], the latter is also propelled simultaneously by the axis of CCR7/CCL21 via a similar mechanism that dendritic cells homing to lymphatic vessels [81, 96]. Additionally, more signaling molecules including VEGF-A [97], platelet-derived growth factor-BB [93], and hepatocyte growth factor [98] had been reported to promote lymphangiogenesis which may also take part in the process of lymphatic metastasis. Kurahara and his coworkers (colleagues) [84] found that high expression of VEGF-C or VEGF-D in the marginal of primary tumor had a significantly higher incidence of lymph node metastasis, whereas the neoplastic lymphatic inside the tumor made no contribution to lymph node metastasis due to its nonfunctional lumen, which is coincident with other reports in PDAC [14, 92, 99]. However, it is still a controversial topic whether tumor induced lymphangiogenesis would promote lymphatic metastasis.

The article "Molecular Mechanism Underlying Lymphatic Metastasis in Pancreatic Cancer" was published in 2014. Journal: Biomed Res Int.

## 4. Microenvironment and Niche

As important as MICs, tumor microenvironment and niche play an essential role in lymphatic metastasis of PDAC. PDAC is a scirrhous and hypoxic tumor, of which the stroma accounts for up to 90% in volume [100]. Growing studies have demonstrated that the extensive interaction between cancer cell and stroma is indispensable in the progression of PDAC. The stroma containing fibroblasts, pancreatic satellite cells, endothelial cells, immune cells, and the extracellular matrix (ECM) creates a dynamic suitable microenvironment and niche for disseminating cancer cells docking and promotes cancer cells growth, invasion, metastasis, and resistance to chemo-/radiotherapy. Severe fibrotic responses is a prominent feature of PDAC; they would exacerbate hypoxia condition within tumor and induce release of a series of cytokines or other mediators like HIF-1, interleukin-8, which not only make for dysplasia of angiogenesis and lymphangiogenesis, but also reversely aggravate the status of desmoplasia and promote MICs formation, finally forming a vicious feedback loop in this evolving process of PDAC [100, 101].

### 4.1. Cancer-Associated Fibroblasts

Cancer-associated fibroblasts (CAFs) are a group of myofibroblasts with a hallmark of contractile properties and alpha-smooth muscle actin (alpha-SMA) staining [100, 102]. As the important component of the hotbed of pancreatic cancer cells, CAFs are significantly associated with the poor prognostic factors including the lymph node status of PDAC and play a pivotal role in progression of PDAC and remolding of tumor microenvironment and niche [100]. Upregulation of alpha-SMA and palladin in fibroblasts induced by the cancer cells containing activated KRAS, the de novo CAFs can promote pancreatic tumorigenesis and progression through their morphologically forming invadopodia-like cellular protrusions which could secrete invadopodia proteins and proteolytic enzymes such as ADAM22, aminopeptidases, and cathepsins D and B used for decomposing the ECM and create an optimum premetastatic niche. Interestingly, they further observed that pancreatic cancers cells (Panc-1 cells) can migrate to distant site following the channel created by the CAFs in the 3D invasion assay [102]. A broad crosstalk between the CAFs and pancreatic cancer cells is important for tumor progression and metastasis. Pancreatic cancer cells and CAFs can interact with each other by releasing various factors to gear up the process of metastasis [103]. Many growth factors produced by cancer cells such as PDGF, TGF-beta, and basic fibroblast growth factor (bFGF) enable fibroblasts to become invasive phenotype of CAFs. Vice versa, the CAFs can also secrete similar growth factors, such as hepatocyte growth factor (HGF), keratinocyte growth factor (KGF), and insulin-like growth factors 1 and 2 (IGF-1 and -2), to stimulate the cancer cells to form malignant phenotype such as MICs. In addition, pancreatic cancer cells could stimulate the CAFs to produce more MMPs such as MMP-2, MMP-7, MMP-9, and MMP-11 which are used for ECM degradation and are conducive for MICs immigrating through the ECM [100, 102, 104].

The article "Molecular Mechanism Underlying Lymphatic Metastasis in Pancreatic Cancer" was published in 2014. Journal: Biomed Res Int.

### 4.2. Pancreatic Stellate Cells

Similar to hepatic stellate cells, pancreatic stellate cells (PSCs) share positive staining of vimentin, desmin, and alpha SMA and store lipid droplets in the cytoplasm, suggesting that they are neither fibroblasts nor smooth muscle cells [100]. PSCs, myofibroblast-like cell activated by cancer cells, and inflammatory factors, such as TNF-alpha, IL-1 and IL-6, PDGF, TGF-beta, FGF, activin A, and reactive oxygen, may facilitate tumor metastatic immigration including lymphatic metastasis. One is secretion of proteolytic matrix-degrading enzymes such as MMPs and another is mass production of matrix and tumor-associated growth factors. Urokinase-type plasminogen activator (uPA) is an important part of tumor stroma. A novel study suggests that uPA and its receptor overexpression were significantly correlated with metastasis of human PDAC. MMP-2 activation and increasing integrin alpha6beta1 expression were observed in a coculture system of fibroblasts and BxPC-3 cells. And finally they proposed that PSCs may have a great role in promoting tumor growth and metastasis via the involvement of uPA-plasminogen cascade [105]. Also, there is evidence in PDAC that MMP-2 activation in conjunction with higher expression of alphaVbeta3 integrin had a significant correlation with lymph node metastasis rather than tumor size, or other prognostic factors [47]. And interestingly, a recent research demonstrated that alphaVbeta3 overexpressed in pancreatic cancer cells can drive lymph node metastases via recruitment of c-Src to the beta3 integrin cytoplasmic tail and triggered series of cascades [48]. In addition, another critical role of PSCs in PDAC progression has been documented to be associated with the pancreatic cancer-stem-cell through enhancing the spheroid-forming ability of cancer cells and inducing the expression of cancer stem cell-related genes ABCG2, Nestin, and LIN28. Therefore, PSCs are considered to be a critical part of the cancer stem cell niche as well [29].

### 4.3. Immunity Response

The abnormal innate or adaptive immunity response in tumor environment or premetastatic sites is thought to be a vital co-conspirator that enables pancreatic cancer cells to survive, grow, and spread to a second anatomic site. In this response, some immune suppressor cells such as CAFs, tolerogenic dendritic cells (DCs), myeloid-derived suppressor cells (MDSCs), immunosuppressive-tumor-associated macrophages, and Treg cells were recruited to play an essential role in lymph node metastasis [106]. In addition, the PSCs expressing Galectin-1 can significantly induce apoptosis of CD4 (+) T cells and CD8 (+) T cells and generation of M2-macrophages, contributing to PSCs-dependent immunoprivilege in the pancreatic cancer milieus [107, 108]. Apart from this, growing evidence indicated that proinflammatory cytokines including interleukin-1 (IL-1), Il-6, IL-11, receptor activator of NF-*κ*B ligand (RANKL, also known as TNFSF11), and TNF*α* play a pivotal role in pancreatic cancer initiation and progression [109]. Lymph nodes, to be worthy of note, as one of the peripheral lymphoid organs of the immune system, are garrisons of B, T, and other immune cells but provide “home” for metastatic cancer cells. However, it is still a pending question about their inner harmonious relationships between immune cells and cancer cells.

### 4.4. Premetastatic Niche

In addition, a new concept of tumor microenvironment, the hypothesis of premetastatic niche, becomes one of the topics that the various fields of oncologists dwell upon with great relish at one time. In a pioneering study, Kaplan et al. [110] noticed that some hematopoietic cells (HPCs) expressing VEGFR1 gathered in predetermined metastatic niche to form cellular clusters ahead of the arrival of tumor cells; moreover, they found that the preferential premetastatic sites of BMDCs clusters formation were distinct in different types of tumor. In a spontaneous animal model of lymphoma, marked VEGFR1+ BMDCs were observed exclusively in the lymph nodes prior to onset of tumor. Further research showed that integrin *α*4*β*1 (also known as VLA-4) expressed in VEGFR1+ cells, when binding with its ligand fibronectin, may facilitate migration of HPCs and circulating inflammatory cells to metastatic niche, and activate VEGFR1+ BMDCs to release various proteinases including MMP-9 in premetastatic niche to destruct basement membranes of ECM to create a conducive microenvironment for engraftment of tumor cells. Moreover, the SDF-1/CXCR4 signal axis could guide BMDCs to the premetastatic niche along with CXCR4+ tumor cells by SDF-1 gradient [16, 78, 110].

The article "Molecular Mechanism Underlying Lymphatic Metastasis in Pancreatic Cancer" was published in 2014. Journal: Biomed Res Int.

Lysyl oxidase (LOX) is an important tumor-secreted factor participating in creating a suitable niche to support disseminated tumor cell growth via promoting formation of a mature ECM and regulating fibronectin activity through FAK activation [111]. LOX cross-linking collagen IV in the basement membrane was essential for recruitment of CD11b+ myeloid cells, which could secrete MMP-2 to resolve collagen to enhance the tumor invasion and recruitment of BMDCs and metastasizing tumor cells to pre-metastatic niche [112]. Endothelial-cells-derived inflammatory chemotaxins S100A8 and S100A9 induced by distant primary tumor may attract Mac1 (macrophage antigen 1) (+)-myeloid cells to the premetastatic site to promote tumor growth in the lung [113]. Exosomes were reported to enhance the metastatic phenotype of primary tumors by educating BMDCs in many cancers [104, 114]. In a rat pancreatic adenocarcinoma model [104], the metastatic ability of cancer cell with CD44v (ASML^wt^) is strikingly stronger than knockdown of CD44v4-v7 (ASML^kd^). Further analysis revealed that functional components of ASML^kd^—soluble fraction, cells, and exosomes were reduced compared to those of ASML^wt^. For instance, CD44v6, c-Met, uPAR, HAsynthase 3 (HAS3), C3, and CD104 were lacking in ASML^kd^ soluble fraction; simultaneously, C-Met, uPAR, and HAS3 expression were also decreased in ASML^kd^ cells, and annexin II, annexin V, heat shock protein 1 (HSP-1), phosphoglycerate kinase 1 (PGK-1), monooxygenase activating protein, and MMP9 were significantly reduced in ASML^kd^ exosomes. And interestingly, the authors observed that ASML^wt^-derived soluble factors could prepare a niche that supports settlement and growth of low metastatic potential ASML^kd^ cells conjunct with exosomes. But the effect on premetastatic niche preparation of exosomes is distinct from that of the soluble fraction; exosomes contain important messages for (pre)metastatic niche preparation, while the soluble fraction may just act as an exosome carrier and/or a reservoir for growth factors, chemokines, and proteases. And finally they proposed that exosomes are the most important factors required for promoting settlement of cancer cells in lymph nodes and lung cooperation with the exosomes carrier soluble matrix, of which the CD44v is essential for promoting leukocyte, stroma, and endothelial cell activation in the (pre)metastatic niche. Another novel study on tumor-derived exosomes led by Peinado pointed out that exosomes could enable bone marrow (BM) progenitors to gain a more pro-metastatic phenotype through the receptor tyrosine kinase MET and also induce vascular leakiness at pre-metastatic sites in melanoma. And importantly, tumor-derived exosomes could recruit BMDCs through upregulating proinflammatory factors at niche. Finally, the authors found that these effects on tumor progression of exosomes could be blocked by one of Ras-related RAB proteins Rab27a [114].

The article "Molecular Mechanism Underlying Lymphatic Metastasis in Pancreatic Cancer" was published in 2014. Journal: Biomed Res Int.

## 5. Implication for Conquering Lymphatic Metastasis of Pancreatic Cancer

Lymphatic metastasis is an “early” event and poor predictor of prognosis in PDAC. Blockade of lymphatic metastasis is as useful as eradication of primary tumor to improve the overall survival for PDAC patients. On the basis of the aforementioned mechanisms, we may endeavor to eliminate lymphatic metastases from early interventions that target both the metastatic seed and soil.

### 5.1. Targeting Cancer Cells

Targeting cancer cells is a quite attractive method; as long as we could eradicate them, everything would be readily resolved, but to be discouraged, still there is no effective and specific drug or means to target cancer cells or metastatic lesion in PDAC. Recently, targeted therapy has been a hot topic especially direct to cancer cells. Hayashi et al. developed a novel strategy for cancer metastasis using a modified strain of *Salmonella typhimurium,* which was administered to both axillary lymph and popliteal lymph node metastases of human pancreatic cancer and fibrosarcoma, respectively, as well as lung metastasis of the fibrosarcoma in nude mice. Strikingly, after 7–21 days of treatment, the metastases were eradicated without chemotherapy or any other treatments, and more importantly, hardly did any adverse effects have been observed [115]. Luo et al. creatively utilized the LyP-1-conjugated nanoparticles for targeting drug delivery to lymphatic metastatic tumors and observed an obvious antitumor effect in mice animal model [116]. ABCG2, as a determining factor of side population, its expression in normal pancreas is absent or low but high in human pancreatic cancer cells. The existing literature implicated hsa-miR-520 h as an important target of ABCG2. Wang and colleagues observed that it resulted in inhibition of cell migration and invasion and decreasing rate of side population cells through transfection of hsa-miR-520 h into Panc-1 cells [30]. MiRNA may therefore be promising as a pancreatic cancer therapy. Although there are a collection of similar experimental results showing an approving effect in PDAC, depressingly, still no one would significantly affect the natural history of PDAC. Accordingly, more in-depth studies are needed to better understand the role of genomics in lymphatic metastasis and design more effective therapies.

The article "Molecular Mechanism Underlying Lymphatic Metastasis in Pancreatic Cancer" was published in 2014. Journal: Biomed Res Int.

### 5.2. Targeting Molecules of Signal Pathways

Signal pathways that have implicated an important role in the initiation and progression of PDAC can be employed as potential therapeutic targets. CXCR-4 is a novel marker for MICs and indicative of aggressive phenotype. Inhibition of the CXCL12/CXCR4 axis is a target for antimetastatic therapy. Saur et al., showed that administration of the selective CXCR4 inhibitor AMD3100 could effectively reduce the enhanced metastatic potential of CXCR4-expressing pancreatic cancer cells [31, 71]. Smad4 deficiency contributes greatly to the invasive phenotype of pancreatic cancer cells. Zhao et al. led a study indicating that suppressing STAT3 expression of Smad4-deficient pancreatic cancer cells could prevent TGFbeta-induced invasion by short hairpin RNA [117]. VEGF/VEGFR is important for angiogenesis, lymphangiogenesis, and vectored lymphatic metastasis in pancreatic cancer. Axitinib, a potent and selective oral inhibitor of VEGFR 1, 2, and 3, plus gemcitabine were reported to have a small, nonstatistically significant benefit for patients with metastatic or locally advanced pancreatic adenocarcinoma in overall survival to gemcitabine alone in an open-label randomized phase II study [118]. Unfortunately, Kindler and colleagues did not observe overall survival benefits for same population between them (median 8.5 versus 8.3 months, resp.) in a double-blind randomized phase III trial [119]. Overall, current targeted drug of signal pathway molecules failed to significantly improve the prognosis for patients with PDAC. Further investigations on developing crucial specific targeted drugs are urgently needed.

The article "Molecular Mechanism Underlying Lymphatic Metastasis in Pancreatic Cancer" was published in 2014. Journal: Biomed Res Int.

### 5.3. Gene Therapy

Gene therapy was first conceptualized by Friedmann and Roblin and meanwhile they raised some cautions against any further attempts at this novel and less-understanding therapy in human patients [120]. Afterwards, this creative therapy gradually transmitted from bench to bedside. The first successful case of curing human gene-defect disease in the United States was performed in 1990 [121]. Cancer as a polygenic disease is accepted by most scholars now. Many scholars attempt to repair the mutation genes or insert a functional gene expressing some antitumor proteins or suicide gene to capture this devastating disease. Therefore, a safe and effective vector of target gene is urgently in need. Vector design has been covered in detail in several recent review articles [122, 123]. Tumor-selective S-TRAIL, a proapoptotic gene, was integrated into stem cell, which was encapsulated by synthetic extracellular matrixes, which was treated for glioblastoma multiforme in mice. And strikingly, it was observed that the engineered stem cells enabled residual tumor cells apoptosis, delayed tumor recurrence, and significantly increased survival of mice [124]. With this in mind, we can modulate the expression of metastasis-related genes in similar method to suppress the metastasis including lymphatic invasion of PDAC. Nevertheless, the applications of gene therapy on cancer remain at a preclinical stage.

### 5.4. Immunotherapy

As early as in the 1950s, the strategy of immunotherapy for cancer has been put forward [125]. And in the past decades, very rapid advances have been made in the researches on tumor immunotherapy, which can be roughly summed up into five categories below: enhancement of innate immune response; construction of specific cancer vaccine (or conjunct with microorganisms) in line with tumor-associated antigens (TAAs), whole-tumor-cell, DNA; monoclonal antibody treatment; adoptive tumor immunotherapy; chimeric antigen receptors. The innate immune response is the key first defense line to tumor cells, enhancement of which is a viable approach to eradicate them undoubtedly. Interleukin 12 (IL12) is a proinflammatory cytokine which can trigger innate and adoptive immunity of the organism by increasing the number of activated macrophages and natural killer cells. A significant antitumor role and hardly any toxic side effects in a murine model of pancreatic cancer were seen via injection of genetically modified fibroblasts expressing IL12 [126]. TRAIL is a death ligand, which can specially induce tumor apoptosis. Studies have provided evidence that TRAIL-overexpressed lymphocytes bundled with the CD3 arm of bispecific antibody EpCAMxCD3, which will insert a significant synergic-specific-antitumor effect, especially targeted cancer stem cell marker EpCAM/ESA in preclinical trial [127, 128]. In addition, a specific tumor-associated antigen would induce immune-specific responses to target tumor cell; hence, to identify more relevant immunogenic targets is urgently needed. At present, several TAAs have been identified in pancreatic cancer such as WT1, MUC1, gastrin, mesothelin, ALDH1A1, annexinA2, SPARC, and KIF20A, which can induce their corresponding specific cytotoxic T lymphocytes to inhibit the tumor growth. However, from all of them, no one is sufficient to combat this tremendous disease, and variant phases of clinical trials are underway to combine immunotherapy with traditional chemotherapy in hope of harvesting more benefits to overall survival.

The article "Molecular Mechanism Underlying Lymphatic Metastasis in Pancreatic Cancer" was published in 2014. Journal: Biomed Res Int.

### 5.5. Subverting Tumor Microenvironments and Niche

Tumor microenvironment and pre(metastatic) site niche provides a receptive “soil” for the “seeds” of MICs or CSCs. Hence, subverting tumor microenvironment and pre(metastatic) site niche may give a novel insight into therapeutic strategy of pancreatic cancer. It is the cardinal hallmark of pancreatic cancer that the desmoplastic hypovascular microenvironment and local hypoxia inside tumor, contribute greatly to the initiation and progression of this disease. Thus, to ameliorate its blood supply and local anoxia inside tumor, alter its status of desmoplasia, as well as reduce the release of the proinflammatory cytokines and production of ECM proteins are no doubt essential strategies to surmount chemoresistance and radiosensitivity. IPI-926, an inhibitor of Hedgehog signaling pathway, can deplete tumor-associated stromal tissue, and it was observed that coadministration with gemcitabine had improved the delivery and efficacy of gemcitabine, obtaining transient stabilization of disease in a mouse model of pancreatic cancer [129]. Similarly, PEGylated human recombinant PH20 hyaluronidase (PEGPH20), which can enzymatically diminish hyaluronan (HA) and induce remodeling of blood vessels inside tumor, rise the delivery of gemcitabine, inhibiting tumor growth and prolonging survival in a genetically engineered mouse model of PDAC [130]. Thus, targeting the tumor stromal microenvironment and pre(metastatic) site niche may be a novel and promising approach for tailored therapies in PDAC.

Unfortunately, little advance has been made in the therapeutic effect for advanced PDAC patients. But these failures should not discourage us from exploring novel treatments for this “incurable” disease. As our understanding of this disease progresses, it would open an avenue for us to discover a novel therapeutic method to conquer the so called “king of carcinoma”.

The article "Molecular Mechanism Underlying Lymphatic Metastasis in Pancreatic Cancer" was published in 2014. Journal: Biomed Res Int.

## 6. Conclusions and Perspectives

The lymph node status has a strong influence on the postoperative long-term survival of patients with pancreatic cancer. Mechanistically, lymphatic metastasis is the concurrent effect of interaction among cancer cells, tumor microenvironment and pre(metastatic) site niche. From putative MICs formation to the subtle alteration of tumor microenvironment and pre/metastatic site niche, from escaping from primary mass to anchoring and adhesion at a new site of lymphatics, and finally a new tumor emerging in lymph node, every step could be deemed as a deliberate machination. The classic hypothesis for tumor metastasis is the “seed-and-soil” hypothesis, which states that cancer cells are the main determinant of tumor spread and the formation of metastasis is the consequence of competitive selection according to the Darwinian model. However, a more likely hypothesis is the “double-reed” style explanation, which underscores a mutual interplay between the cancer cell and its surroundings. On the one hand, the microenvironment can inform the invasive phenotype of cancer cells and release some signal molecules to direct MICs toward the adaptive site; on the other hand, cancer cells can direct stromal cells, myeloid-derived cells, and associated chemokines to tumor surrounding and premetastatic niches to reform an environment well suited for tumor growth and metastasis.

Of note, the inclination for lymphatic metastasis in PDAC is possibly and mainly based on three factors: first, the CXCR-4 expressed in cancer cells indicates a metastatic phenotype and simultaneously SDF-1/CXCR-4 promotes the movement of MICs toward lymph nodes; second, the VEGF-D/C/VEGFR-3 initiates lymphangiogenesis and VEGF-D/C plays a role in chemotaxis for new/existed lymphatics expressing VEGFR-3; and third, CCL21/CCR7 induces host immune tolerance to tumor cells at the metastatic site, and concomitantly, CCL21 drives tumor cells expressing CCR7 toward lymphatic vessels in a pattern of the concentration gradient. However, yet many open questions should be resolved that whether tumor cells are transported by lymph nodes passively or actively, whether the lymph nodes promote systemic spread of the tumor cells by serving as a reservoir, and whether tumor cells enable lymph nodes to be a favorable microenvironment for metastases maturation. Therefore, a better understanding of these critical aspects for lymphatic metastasis of PDAC will open a new avenue for ameliorating the abysmal prognosis.

The article "Molecular Mechanism Underlying Lymphatic Metastasis in Pancreatic Cancer" was published in 2014. Journal: Biomed Res Int.

## Figures and Tables

**Figure 1:** Lymphatic metastasis in PDAC: it is not a monodrama. Lymphatic metastasis is the concurrent effect of interaction among cancer cells, tumor microenvironment, and premetastatic site niche. The role of evolution of cancer cell and microenvironment in this abysmal biologic process is performed in a “double-reed” style. Under the influence of fertile microenvironment and accumulating gene alterations (KRAS, SMAD4, TP53+, Ink4a/Arf, etc.), a normal pancreatic epithelial cell underwent the long processes such as “acinar-to-ductal metaplasia” and “epithelia-mesenchymal transition” and finally sequentially forming a metastasis-initiating cell, which could initiate lymphatic metastasis under the guidance of specific chemokines (SDF-1, CCL19/CCL21, VEGF-C/D, etc.). Accordingly, potential therapeutic strategies targeted to the lymphatic metastasis of pancreatic cancer include: (1) targeting cancer cells (CSCs, MICs), (2) targeting molecules of signal pathways to the tumor, and (3) subverting the tumor microenvironments and niche.

**Figure 2:** Establishment of a highly lymphatic metastatic subline BxPC-3-LN including 5 steps: (1) subcutaneous footpad injection of nude mice with BxPC-3 cells; (2) doing autopsy to remove the possible metastatic lymph nodes which were confirmed by pathological confirmation; (3) isolation of metastatic cancer cells from identified lymph nodes; (4) selection and subculture of cells; (5) reinjection in nude mice for additional rounds and finally obtaining desired cell line BxPC-3-LN. And in the end, further analysis of two cell lines is urgently required such as comparison of gene and miRNAs expression profile via microarray.

**Table 1:** Markers of cancer stem cells in pancreatic cancer.

Cancer stem cells	Markers	References
Tumor-initiating population	EpCAM/ESA^+^CD44^+^CD24^+^	[11, 13]
	CD133^+^	[11, 13]
	ALDH-1^+^	[11, 28]
	Side population/ABCG2	[29, 30]
Metastasis-initiating cells	CD133^+^CXCR-4^+^	[9, 31]

**Table 2:** Metastasis-related miRNAs in pancreatic cancer.

miRNA	Impact on metastatic processes	Target genes	References
miR-146a/b	Suppressing	EGFR, IRAK-1, MMP16, and NF-*κ*B	[61]
let-7 family	Suppressing	HMGA2, MYC, NOTCH, RAS, COL1A2, MT1-MMP, MMP-14	[62]
miR-141, and miR-200a/b/c, miR-429	Suppressing	ZEB1, ZEB2, E-CADHERIN, N-CADHERIN	[38]
miR-34 family	Suppressing	NOTCH, BCL-2, NANOG, SOX2, and N-MYC	[39]
miR-20a	Suppressing	STAT3	[63]
miR-126	Suppressing	ADAM9	[64]
miR-150	Suppressing	MUC4	[36]
miR-30 family	Suppressing	VIMENTIN and SNAIL-1	[65]
miR-143/145	Suppressing	KRAS, RREB1	[34]
miR-486	Promoting	CD40	[66]
miR-224	Promoting	CD40	[66]
miR-10a, miR-10b	Promoting	HOXA1, HOXB1, and HOXB3	[40, 41]
miRNA-27a	Promoting	SPRY2	[42]

The article "Molecular Mechanism Underlying Lymphatic Metastasis in Pancreatic Cancer" was published in 2014. Journal: Biomed Res Int.

## References

[1] Vincent A, Herman J, Schulick R, Hruban RH, Goggins M (2011). Pancreatic cancer. *The Lancet*.

[2] Slidell MB, Chang DC, Cameron JL (2008). Impact of total lymph node count and lymph node ratio on staging and survival after pancreatectomy for pancreatic adenocarcinoma: a large, population-based analysis. *Annals of Surgical Oncology*.

[3] Furukawa H, Okada S, Saisho H (1996). Clinicopathologic features of small pancreatic adenocarcinoma. A collective study. *Cancer*.

[4] Hosch SB, Knoefel WT, Metz S (1997). Early lymphatic tumor cell dissemination in pancreatic cancer: frequency and prognostic significance. *Pancreas*.

[5] Demeure MJ, Doffek KM, Komorowski RA (1998). Adenocarcinoma of the pancreas: detection of occult metastases in regional lymph nodes by a polymerase chain reaction-based assay. *Cancer*.

[6] Ando N, Nakao A, Nomoto S (1997). Detection of mutant K-ras in dissected paraaortic lymph nodes of patients with pancreatic adenocarcinoma. *Pancreas*.

[7] Achen MG, Stacker SA (2008). Molecular control of lymphatic metastasis. *Annals of the New York Academy of Sciences*.

[8] Rosen JM, Jordan CT (2009). The increasing complexity of the cancer stem cell paradigm. *Science*.

[9] Hermann PC, Huber SL, Herrler T (2007). Distinct populations of cancer stem cells determine tumor growth and metastatic activity in human pancreatic cancer. *Cell Stem Cell*.

[10] Brabletz T, Jung A, Spaderna S, Hlubek F, Kirchner T (2005). Migrating cancer stem cells—an integrated concept of malignant tumour progression. *Nature Reviews Cancer*.

[11] Ni X, Long J, Cen P (2011). Pancreatic cancer tumor initiating cells: the molecular regulation and therapeutic values. *Journal of Cellular and Molecular Medicine*.

[12] Bonnet D, Dick JE (1997). Human acute myeloid leukemia is organized as a hierarchy that originates from a primitive hematopoietic cell. *Nature Medicine*.

[13] Li C, Heidt DG, Dalerba P (2007). Identification of pancreatic cancer stem cells. *Cancer Research*.

[14] Maeda S, Shinchi H, Kurahara H (2008). CD133 expression is correlated with lymph node metastasis and vascular endothelial growth factor-C expression in pancreatic cancer. *British Journal of Cancer*.

[15] Ishizawa K, Rasheed ZA, Karisch R (2010). Tumor-initiating cells are rare in many human tumors. *Cell Stem Cell*.

[16] Cui K, Zhao W, Wang C (2011). The CXCR4-CXCL12 pathway facilitates the progression of pancreatic cancer via induction of angiogenesis and lymphangiogenesis. *Journal of Surgical Research*.

[17] Singh S, Srivastava SK, Bhardwaj A, Owen LB, Singh AP (2010). CXCL12-CXCR4 signalling axis confers gemcitabine resistance to pancreatic cancer cells: a novel target for therapy. *British Journal of Cancer*.

The article "Molecular Mechanism Underlying Lymphatic Metastasis in Pancreatic Cancer" was published in 2014. Journal: Biomed Res Int.

[18] Li R, Sonik A, Stindl R, Rasnick D, Duesberg P (2000). Aneuploidy versus gene mutation hypothesis of cancer: recent study claims mutation but is found to support aneuploidy. *Proceedings of the National Academy of Sciences of the United States of America*.

[19] Wu C, Miao X, Huang L (2012). Genome-wide association study identifies five loci associated with susceptibility to pancreatic cancer in Chinese populations. *Nature Genetics*.

[20] Long J, Luo G, Liu C (2012). Development of a unique mouse model for pancreatic cancer lymphatic metastasis. *International Journal of Oncology*.

[21] Aguirre AJ, Bardeesy N, Sinha M (2003). Activated Kras and Ink4a/Arf deficiency cooperate to produce metastatic pancreatic ductal adenocarcinoma. *Genes and Development*.

[22] Hingorani SR, Wang L, Multani AS (2005). Trp53R172H and KrasG12D cooperate to promote chromosomal instability and widely metastatic pancreatic ductal adenocarcinoma in mice. *Cancer Cell*.

[23] Morton JP, Timpson P, Karim SA (2010). Mutant p53 drives metastasis and overcomes growth arrest/senescence in pancreatic cancer. *Proceedings of the National Academy of Sciences of the United States of America*.

[24] Yachida S, Jones S, Bozic I (2010). Distant metastasis occurs late during the genetic evolution of pancreatic cancer. *Nature*.

[25] Campbell PJ, Yachida S, Mudie LJ (2010). The patterns and dynamics of genomic instability in metastatic pancreatic cancer. *Nature*.

[26] Kim HN, Choi DW, Lee KT (2007). Gene expression profiling in lymph node-positive and lymph node-negative pancreatic cancer. *Pancreas*.

[27] Nakamura T, Furukawa Y, Nakagawa H (2004). Genome-wide cDNA microarray analysis of gene expression profiles in pancreatic cancers using populations of tumor cells and normal ductal epithelial cells selected for purity by laser microdissection. *Oncogene*.

[28] Visus C, Wang Y, Lozano-Leon A (2011). Targeting ALDHbright human carcinoma-initiating cells with ALDH1A1-specific CD8+ T cells. *Clinical Cancer Research*.

[29] Hamada S, Masamune A, Takikawa T (2012). Pancreatic stellate cells enhance stem cell-like phenotypes in pancreatic cancer cells. *Biochemical and Biophysical Research Communications*.

[30] Wang F, Xue X, Wei J (2010). Hsa-miR-520h downregulates ABCG2 in pancreatic cancer cells to inhibit migration, invasion, and side populations. *British Journal of Cancer*.

[31] Marchesi F, Monti P, Leone BE (2004). Increased survival, proliferation, and migration in metastatic human pancreatic tumor cells expressing functional CXCR4. *Cancer Research*.

[32] Calin GA, Croce CM (2006). MicroRNA signatures in human cancers. *Nature Reviews Cancer*.

The article "Molecular Mechanism Underlying Lymphatic Metastasis in Pancreatic Cancer" was published in 2014. Journal: Biomed Res Int.

[33] Tavano F, di Mola FF, Piepoli A (2012). Changes in miR-143 and miR-21 expression and clinicopathological correlations in pancreatic cancers. *Pancreas*.

[34] Kent OA, Chivukula RR, Mullendore M (2010). Repression of the miR-143/145 cluster by oncogenic Ras initiates a tumor-promoting feed-forward pathway. *Genes and Development*.

[35] Yu S, Lu Z, Liu C (2010). miRNA-96 suppresses KRAS and functions as a tumor suppressor gene in pancreatic cancer. *Cancer Research*.

[36] Srivastava SK, Bhardwaj A, Singh S (2011). MicroRNA-150 directly targets MUC4 and suppresses growth and malignant behavior of pancreatic cancer cells. *Carcinogenesis*.

[37] Choudhury A, Moniaux N, Ulrich AB (2004). MUC4 mucin expression in human pancreatic tumours is affected by organ environment: the possible role of TGF*β*2. *British Journal of Cancer*.

[38] Wellner U, Schubert J, Burk UC (2009). The EMT-activator ZEB1 promotes tumorigenicity by repressing stemness-inhibiting microRNAs. *Nature Cell Biology*.

[39] Ji Q, Hao X, Zhang M (2009). MicroRNA miR-34 inhibits human pancreatic cancer tumor-initiating cells. *PLoS ONE*.

[40] Ohuchida K, Mizumoto K, Lin C (2012). MicroRNA-10a is overexpressed in human pancreatic cancer and involved in its invasiveness partially via suppression of the HOXA1 gene. *Annals of Surgical Oncology*.

[41] Weiss FU, Marques IJ, Woltering JM (2009). Retinoic acid receptor antagonists inhibit miR-10a expression and block metastatic behavior of pancreatic cancer. *Gastroenterology*.

[42] Ma Y, Yu S, Zhao W, Lu Z, Chen J (2010). MiR-27a regulates the growth, colony formation and migration of pancreatic cancer cells by targeting Sprouty2. *Cancer Letters*.

[43] Drabsch Y, Ten DP (2012). TGF-beta signalling and its role in cancer progression and metastasis. *Cancer and Metastasis Reviews*.

[44] Wang P, Fan J, Chen Z (2009). Low-level expression of Smad7 correlates with lymph node metastasis and poor prognosis in patients with pancreatic cancer. *Annals of Surgical Oncology*.

[45] Jiang H, He C, Geng S (2012). RhoT1 and Smad4 are correlated with lymph node metastasis and overall survival in pancreatic cancer. *PLoS ONE*.

[46] Kabashima A, Higuchi H, Takaishi H (2009). Side population of pancreatic cancer cells predominates in TGF-*β*-mediated epithelial to mesenchymal transition and invasion. *International Journal of Cancer*.

[47] Hosotani R, Kawaguchi M, Masui T (2002). Expression of integrin alphaVbeta3 in pancreatic carcinoma: relation to MMP-2 activation and lymph node metastasis. *Pancreas*.

[48] Desgrosellier JS, Barnes LA, Shields DJ (2009). An integrin *α* v *Β* 3-c-Src oncogenic unit promotes anchorage-independence and tumor progression. *Nature Medicine*.

The article "Molecular Mechanism Underlying Lymphatic Metastasis in Pancreatic Cancer" was published in 2014. Journal: Biomed Res Int.

[49] Dai J, Ai K, Du Y, Chen G (2011). Sonic hedgehog expression correlates with distant metastasis in pancreatic adenocarcinoma. *Pancreas*.

[50] Eberl M, Klingler S, Mangelberger D (2012). Hedgehog-EGFR cooperation response genes determine the oncogenic phenotype of basal cell carcinoma and tumour-initiating pancreatic cancer cells. *EMBO Molecular Medicine*.

[51] Joost S, Almada LL, Rohnalter V (2012). GLI1 inhibition promotes epithelial-to-mesenchymal transition in pancreatic cancer cells. *Cancer Research*.

[52] Bailey JM, Swanson BJ, Hamada T (2008). Sonic hedgehog promotes desmoplasia in pancreatic cancer. *Clinical Cancer Research*.

[53] Lai EC (2004). Notch signaling: control of cell communication and cell fate. *Development*.

[54] Mullendore ME, Koorstra J-B, Li Y-M (2009). Ligand-dependent notch signaling is involved in tumor initiation and tumor maintenance in pancreatic cancer. *Clinical Cancer Research*.

[55] Chen H-T, Cai Q-C, Zheng J-M (2012). High expression of delta-like ligand 4 predicts poor prognosis after curative resection for pancreatic cancer. *Annals of Surgical Oncology*.

[56] Bao B, Wang Z, Ali S (2011). Notch-1 induces epithelial-mesenchymal transition consistent with cancer stem cell phenotype in pancreatic cancer cells. *Cancer Letters*.

[57] Sureban SM, May R, Lightfoot SA (2011). DCAMKL-1 regulates epithelial-mesenchymal transition in human pancreatic cells through a miR-200a-dependent mechanism. *Cancer Research*.

[58] Hanlon L, Avila JL, Demarest RM (2010). Notch1 functions as a tumor suppressor in a model of K-ras-induced pancreatic ductal adenocarcinoma. *Cancer Research*.

[59] De La O J-P, Emerson LL, Goodman JL (2008). Notch and Kras reprogram pancreatic acinar cells to ductal intraepithelial neoplasia. *Proceedings of the National Academy of Sciences of the United States of America*.

[60] De La O J-P, Murtaugh LC (2009). Notch and Kras in pancreatic cancer: at the crossroads of mutation, differentiation and signaling. *Cell Cycle*.

[61] Li Y, VandenBoom TG, Wang Z (2010). miR-146a suppresses invasion of pancreatic cancer cells. *Cancer Research*.

[62] Dangi-Garimella S, Strouch MJ, Grippo PJ, Bentrem DJ, Munshi HG (2011). Collagen regulation of let-7 in pancreatic cancer involves TGF-*β*1-mediated membrane type 1-matrix metalloproteinase expression. *Oncogene*.

[63] Yan H, Wu J, Liu W (2010). MicroRNA-20a overexpression inhibited proliferation and metastasis of pancreatic carcinoma cells. *Human Gene Therapy*.

[64] Hamada S, Satoh K, Fujibuchi W (2012). MiR-126 acts as a tumor suppressor in pancreatic cancer cells via the regulation of ADAM9. *Molecular Cancer Research*.

The article "Molecular Mechanism Underlying Lymphatic Metastasis in Pancreatic Cancer" was published in 2014. Journal: Biomed Res Int.

[65] Joglekar MV, Patil D, Joglekar VM (2009). The miR-30 family microRNAs confer epithelial phenotype to human pancreatic cells. *Islets*.

[66] Mees ST, Mardin WA, Sielker S (2009). Involvement of CD40 targeting miR-224 and miR-486 on the progression of pancreatic ductal adenocarcinomas. *Annals of Surgical Oncology*.

[67] Li X, Ma Q, Xu Q (2012). SDF-1/CXCR4 signaling induces pancreatic cancer cell invasion and epithelial-mesenchymal transition in vitro through non-canonical activation of Hedgehog pathway. *Cancer Letters*.

[68] Mimeault M, Batra SK (2008). Recent progress on normal and malignant pancreatic stem/progenitor cell research: therapeutic implications for the treatment of type 1 or 2 diabetes mellitus and aggressive pancreatic cancer. *Gut*.

[69] Wang Z, Ma Q, Liu Q (2008). Blockade of SDF-1/CXCR4 signalling inhibits pancreatic cancer progression in vitro via inactivation of canonical Wnt pathway. *British Journal of Cancer*.

[70] Thomas RM, Kim J, Revelo-Penafiel MP, Angel R, Dawson DW, Lowy AM (2008). The chemokine receptor CXCR4 is expressed in pancreatic intraepithelial neoplasia. *Gut*.

[71] Saur D, Seidler B, Schneider G (2005). CXCR4 expression increases liver and lung metastasis in a mouse model of pancreatic cancer. *Gastroenterology*.

[72] Liu F, Lang R, Wei J (2009). Increased expression of SDF-1/CXCR4 is associated with lymph node metastasis of invasive micropapillary carcinoma of the breast. *Histopathology*.

[73] Chang S-C, Lin P-C, Yang S-H, Wang H-S, Li AF-Y, Lin J-K (2009). SDF-1*α* G801A polymorphism predicts lymph node metastasis in stage T3 colorectal cancer. *Annals of Surgical Oncology*.

[74] Zhao B-C, Wang Z-J, Mao W-Z (2011). CXCR4/SDF-1 axis is involved in lymph node metastasis of gastric carcinoma. *World Journal of Gastroenterology*.

[75] Shen X, Artinyan A, Jackson D, Thomas RM, Lowy AM, Kim J (2010). Chemokine receptor CXCR4 enhances proliferation in pancreatic cancer cells through akt and erk dependent pathways. *Pancreas*.

[76] Lee Y, Kim SJ, Park HD (2010). PAUF functions in the metastasis of human pancreatic cancer cells and upregulates CXCR4 expression. *Oncogene*.

[77] Lee Y, Kim SJ, Min HJ, Jo JY, Park EH, Koh SS (2011). PAUF promotes adhesiveness of pancreatic cancer cells by modulating focal adhesion kinase. *Experimental and Molecular Medicine*.

[78] Chen Z, Chen LY, Wang P (2012). Tumor microenvironment varies under different TCM ZHENG models and correlates with treatment response to herbal medicine. *Evidence-Based Complementary and Alternative Medicine*.

[79] Mori T, Doi R, Koizumi M (2004). CXCR4 antagonist inhibits stromall cell-derived factor 1-induced migration and invasion of human pancreatic cancer. *Molecular Cancer Therapeutics*.

The article "Molecular Mechanism Underlying Lymphatic Metastasis in Pancreatic Cancer" was published in 2014. Journal: Biomed Res Int.

[80] Issa A, Le TX, Shoushtari AN, Shields JD, Swartz MA (2009). Vascular endothelial growth factor-C and C-C chemokine receptor 7 in tumor cell-lymphatic cross-talk promote invasive phenotype. *Cancer Research*.

[81] Sperveslage J, Frank S, Heneweer C (2012). Lack of CCR7 expression is rate limiting for lymphatic spread of pancreatic ductal adenocarcinoma. *International Journal of Cancer*.

[82] Shields JD, Fleury ME, Yong C, Tomei AA, Randolph GJ, Swartz MA (2007). Autologous chemotaxis as a mechanism of tumor cell homing to lymphatics via interstitial flow and autocrine CCR7 signaling. *Cancer Cell*.

[83] Emmett MS, Lanati S, Dunn DBA, Stone OA, Bates DO (2011). CCR7 mediates directed growth of melanomas towards lymphatics. *Microcirculation*.

[84] Kurahara H, Takao S, Maemura K, Shinchi H, Natsugoe S, Aikou T (2004). Impact of vascular endothelial growth factor-C and -D expression in human pancreatic cancer: its relationship to lymph node metastasis. *Clinical Cancer Research*.

[85] Joukov V, Sorsa T, Kumar V (1997). Proteolytic processing regulates receptor specificity and activity of VEGF-C. *The EMBO Journal*.

[86] Stacker SA, Stenvers K, Caesar C (1999). Biosynthesis of vascular endothelial growth factor-D involves proteolytic processing which generates non-covalent homodimers. *Journal of Biological Chemistry*.

[87] He Y, Rajantie I, Pajusola K (2005). Vascular endothelial cell growth factor receptor 3-mediated activation of lymphatic endothelium is crucial for tumor cell entry and spread via lymphatic vessels. *Cancer Research*.

[88] Smith NR, Baker D, James NH (2010). Vascular endothelial growth factor receptors VEGFR-2 and VEGFR-3 are localized primarily to the vasculature in human primary solid cancers. *Clinical Cancer Research*.

[89] Kaplan RN, Psaila B, Lyden D (2006). Bone marrow cells in the “pre-metastatic niche”: within bone and beyond. *Cancer and Metastasis Reviews*.

[90] Tang RF, Itakura J, Aikawa T (2001). Overexpression of lymphangiogenic growth factor VEGF-C in human pancreatic cancer. *Pancreas*.

[91] Alitalo K, Carmeliet P (2002). Molecular mechanisms of lymphangiogenesis in health and disease. *Cancer Cell*.

[92] Schneider M, Büchler P, Giese N (2006). Role of lymphangiogenesis and lymphangiogenic factors during pancreatic cancer progression and lymphatic spread. *International Journal of Oncology*.

[93] Cao R, Björndahl MA, Religa P (2004). PDGF-BB induces intratumoral lymphangiogenesis and promotes lymphatic metastasis. *Cancer Cell*.

[94] Lee K, Park DJ, Choe G, Kim HH, Kim WH, Lee HS (2010). Increased intratumoral lymphatic vessel density correlates with lymph node metastasis in early gastric carcinoma. *Annals of Surgical Oncology*.

The article "Molecular Mechanism Underlying Lymphatic Metastasis in Pancreatic Cancer" was published in 2014. Journal: Biomed Res Int.

[95] Otto N, Schulz P, Scholz A (2012). The proline TP53 variant stimulates likely lymphangiogenesis in an orthotopic mouse model of pancreatic cancer. *British Journal of Cancer*.

[96] Nakata B, Fukunaga S, Noda E, Amano R, Yamada N, Hirakawa K (2008). Chemokine receptor CCR7 expression correlates with lymph node metastasis in pancreatic cancer. *Oncology*.

[97] Wuest TR, Carr DJJ (2010). VEGF-A expression by HSV-1-infected cells drives corneal lymphangiogenesis. *Journal of Experimental Medicine*.

[98] Saito Y, Nakagami H, Morishita R (2006). Transfection of human hepatocyte growth factor gene ameliorates secondary lymphedema via promotion of lymphangiogenesis. *Circulation*.

[99] Tang R-F, Wang S-X, Peng L (2006). Expression of vascular endothelial growth factors A and C in human pancreatic cancer. *World Journal of Gastroenterology*.

[100] Luo G, Long J, Zhang B (2012). Stroma and pancreatic ductal adenocarcinoma: an interaction loop. *Biochimica et Biophysica Acta*.

[101] Hussain F, Wang J, Ahmed R (2010). The expression of IL-8 and IL-8 receptors in pancreatic adenocarcinomas and pancreatic neuroendocrine tumours. *Cytokine*.

[102] Brentnall TA, Lai LA, Coleman J, Bronner MP, Pan S, Chen R (2012). Arousal of cancer-associated stroma: overexpression of palladin activates fibroblasts to promote tumor invasion. *PLoS ONE*.

[103] Algül H, Treiber M, Lesina M, Schmid RM (2007). Mechanisms of disease: chronic inflammation and cancer in the pancreas—a potential role for pancreatic stellate cells?. *Nature Clinical Practice Gastroenterology and Hepatology*.

[104] Jung T, Castellana D, Klingbeil P (2009). CD44v6 dependence of premetastatic niche preparation by exosomes. *Neoplasia*.

[105] He Y, Liu X-D, Chen Z-Y (2007). Interaction between cancer cells and stromal fibroblasts is required for activation of the uPAR-uPA-MMP-2 cascade in pancreatic cancer metastasis. *Clinical Cancer Research*.

[106] Yamato I, Sho M, Nomi T (2009). Clinical importance of B7-H3 expression in human pancreatic cancer. *British Journal of Cancer*.

[107] DeNardo DG, Barreto JB, Andreu P (2009). CD4(+) T cells regulate pulmonary metastasis of mammary carcinomas by enhancing protumor properties of macrophages. *Cancer Cell*.

[108] Qian B-Z, Pollard JW (2010). Macrophage diversity enhances tumor progression and metastasis. *Cell*.

[109] Li N, Grivennikov SI, Karin M (2011). The unholy trinity: inflammation, cytokines, and STAT3 shape the cancer microenvironment. *Cancer Cell*.

[110] Kaplan RN, Riba RD, Zacharoulis S (2005). VEGFR1-positive haematopoietic bone marrow progenitors initiate the pre-metastatic niche. *Nature*.

The article "Molecular Mechanism Underlying Lymphatic Metastasis in Pancreatic Cancer" was published in 2014. Journal: Biomed Res Int.

[111] Erler JT, Bennewith KL, Nicolau M (2006). Lysyl oxidase is essential for hypoxia-induced metastasis. *Nature*.

[112] Erler JT, Bennewith KL, Cox TR (2009). Macrophage diversity enhances tumor progression and metastasis. *Cancer Cell*.

[113] Hiratsuka S, Watanabe A, Aburatani H, Maru Y (2006). Tumour-mediated upregulation of chemoattractants and recruitment of myeloid cells predetermines lung metastasis. *Nature Cell Biology*.

[114] Peinado H, Aleckovic M, Lavotshkin S (2012). Melanoma exosomes educate bone marrow progenitor cells toward a pro-metastatic phenotype through MET. *Nature Medicine*.

[115] Hayashi K, Zhao M, Yamauchi K (2009). Cancer metastasis directly eradicated by targeted therapy with a modified Salmonella typhimurium. *Journal of Cellular Biochemistry*.

[116] Luo G, Yu X, Jin C (2010). LyP-1-conjugated nanoparticles for targeting drug delivery to lymphatic metastatic tumors. *International Journal of Pharmaceutics*.

[117] Zhao S, Venkatasubbarao K, Lazor JW (2008). Inhibition of STAT3Tyr705 phosphorylation by Smad4 suppresses transforming growth factor *β*-mediated invasion and metastasis in pancreatic cancer cells. *Cancer Research*.

[118] Spano J-P, Chodkiewicz C, Maurel J (2008). Efficacy of gemcitabine plus axitinib compared with gemcitabine alone in patients with advanced pancreatic cancer: an open-label randomised phase II study. *The Lancet*.

[119] Kindler HL, Ioka T, Richel DJ (2011). Axitinib plus gemcitabine versus placebo plus gemcitabine in patients with advanced pancreatic adenocarcinoma: a double-blind randomised phase 3 study. *The Lancet Oncology*.

[120] Friedmann T, Roblin R (1972). Gene therapy for human genetic disease?. *Science*.

[121] Blaese RM, Culver KW, Miller AD (1995). T lymphocyte-directed gene therapy for ADA- SCID: initial trial results after 4 years. *Science*.

[122] Mukherjee S, Thrasher AJ (2011). Progress and prospects: advancements in retroviral vector design, generation, and application. *Human Gene Therapy*.

[123] Dong JY, Woraratanadharm J (2005). Gene therapy vector design strategies for the treatment of cancer. *Future Oncology*.

[124] Kauer TM, Figueiredo J-L, Hingtgen S, Shah K (2012). Encapsulated therapeutic stem cells implanted in the tumor resection cavity induce cell death in gliomas. *Nature Neuroscience*.

[125] Delouys F (1953). Biological treatment of cancer. *Le Scalpel*.

[126] Péron JM, Bureau C, Gourdy P (2007). Treatment of experimental murine pancreatic peritoneal carcinomatosis with fibroblasts genetically modified to express IL12: a role for peritoneal innate immunity. *Gut*.

The article "Molecular Mechanism Underlying Lymphatic Metastasis in Pancreatic Cancer" was published in 2014. Journal: Biomed Res Int.

[127] Cioffi M, Dorado J, Baeuerle PA, Heeschen C (2012). EpCAM/CD3-bispecific T-cell engaging antibody MT110 eliminates primary human pancreatic cancer stem cells. *Clinical Cancer Research*.

[128] Groth A, Salnikov AV, Ottinger S (2012). New gene-immunotherapy combining TRAIL-lymphocytes and EpCAMxCD3 bispecific antibody for tumor targeting. *Clinical Cancer Research*.

[129] Olive KP, Jacobetz MA, Davidson CJ (2009). Inhibition of Hedgehog signaling enhances delivery of chemotherapy in a mouse model of pancreatic cancer. *Science*.

[130] Jacobetz MA, Chan DS, Neesse A (2012). Hyaluronan impairs vascular function and drug delivery in a mouse model of pancreatic cancer. *Gut*.

